The article "Using of artificial neural networks and different evolutionary algorithms to predict the viscosity and thermal conductivity of silica-alumina-MWCN/water nanofluid" was retracted in 2025. Reasons: unreliable results or conclusions; concerns about the authorship.

# Using of artificial neural networks and different evolutionary algorithms to predict the viscosity and thermal conductivity of silica-alumina-MWCN/water nanofluid

**DOI:** 10.1016/j.heliyon.2024.e26279

**Published:** 2024-02-10

**Authors:** Mohammadreza Baghoolizadeh, Dheyaa J. Jasim, S. Mohammad Sajadi, Reza Rostamzadeh- Renani, Mohammad Rostamzadeh- Renani, Maboud Hekmatifar

**Affiliations:** a Department of Mechanical Engineering, Shahrekord University, Shahrekord 88186-34141, Iran; b Department of Petroleum Engineering, Al-Amarah University College, Maysan, Iraq; c Department of Nutrition, Cihan University-Erbil, Kurdistan Region, Iraq; d Energy Department, Politecnico di Milano, Via Lambruschini 4, 20156 Milan, Italy; e Department of mechanical engineering, Khomeinishahr branch, Islamic Azad University, Khomeinishahr, Iran

**Keywords:** Meta-heuristic, NSGA II, Correlation coefficient, Nanofluid, Pareto front

## Abstract

This study predicts the parameters such as viscosity and thermal conductivity in silica-alumina-MWCN/water nanofluid using the artificial intelligence method and using design variables such as solid volume fraction and temperature. In this study, 6 optimization algorithms were used to predict and numerically model the μ_nf_ and TC of silica-alumina-MWCNT/water–NF. In this study, six measurement criteria were used to evaluate the estimates obtained from the coupling process of GMDH ANN with each of these 6 optimization algorithms. The results reveal that the influence of the φ is notably higher on both μ_nf_ and TC with values of 0.83 for μ_nf_ and 0.92 for TC, while Temp has a relatively weaker impact with −0.5 for μ_nf_ and 0.38 for TC. Among various algorithms, the coupling of the evolutionary algorithm NSGA II with ANN and GMDH performs best in predicting μ_nf_ and TC for the NF, with a maximum margin of deviation of −0.108 and an R^2^ evaluation criterion of 0.99996 for μ_nf_ and 1 for TC, indicating exceptional model accuracy. In the subsequent phase, a meta-heuristic Genetic Algorithm minimizes μ_nf_ and TC values. Four points (A, B, C, and D) along the Pareto front are selected, with point A representing the optimal state characterized by low values of φ and Temp (0.0002 and 50.8772, respectively) and corresponding target function values of 0.9988 for μ_nf_ and 0.6344 for TC. In contrast, point D represents the highest values of φ and Temp (0.49986 and 59.9775, respectively) and yields target function values of 2.382 for μ_nf_ and 0.8517 for TC. This analysis aids in identifying the optimal operating conditions for maximizing NF performance.

## Nomenclature

μ_nf_: Viscosity
TC: Thermal Conductivity
φ: Solid Volume Fraction

**Abbreviation**
Temp: Temperature
RB: Rheological behavior
NFs: Nanofluids
NPs: Nanoparticles
MOD: Margin of Deviation
MSE: Mean square error
MAE: Average absolute error
MAPE: Mean absolute percentage error
RMSE: Root Mean Square Error
R: Correlation Coefficient
R^2^: R-Squared
MLP: Multi-Layer Perceptron
GMDH: Group Method of Data Handling
MOPSO: Multi-Objective Particle Swarm Optimization
MALO: Multi objective Ant Lion Optimization Algorithm
MOMFO: Multi objective Moth Flame Optimization Algorithm
MOWOA: Multi-objective whale optimization Algo
MOGOA: Multi objective Grasshopper Optimization Algorithm
NSGA-II: Non-Dominated Sorted Genetic Algo

## 1 Introduction

Natural heat transfer in liquids is an important phenomenon in engineering and industries with wide applications in various fields, such as cooling fluids in heating systems. Common fluids such as water, ethylene glycol (EG), and lubricant are used in the cooling process of the equipment, and heat is transferred by these fluids. However, there is a fundamental problem: fluids have a lower TC than solids. To solve this problem, researchers decided to provide new methods for the TC of these fluids. The first idea in this field was the plan of dispersing metal particles in the base fluid. This plan, which Maxwell presented, has problems such as settling and agglomeration of particles and blocking pipes, which causes a lot of energy loss [1]. However, the advancement of the technology of making particles on a nanoscale solved this issue to a large extent [[2], [3], [4]]. NF technology is an interdisciplinary science that has had a significant development in nanoscience, nanotechnology and thermal engineering in the past decades. The purpose of making NF is to obtain higher thermal properties and lower pumping power to make a stable suspension. It is worth noting that these particles have a TC up to hundreds of times higher than the base fluid, so it is expected that by adding these particles with a scale of 1 nm–100 nm to the base fluid, the TC of base fluids will increase significantly [[5], [6], [7]]. Today, various experiments were conducted in the field of the effect of NPs on TC and μ_nf_ [8]. These tests are based on the investigation of some effective factors such φ, Temp, pH of the suspension, the size of NPs, the mechanisms of heat transfer in NFs, including Brownian motion, etc., on the rheological properties of NFs. Some of these researches are discussed below [[9], [10], [11], [12]]. In the study by Chu et al. [13], the RB of MWCNT-TiO_2_/5W40 hybrid NF was investigated. This study is based on two experimental methods and regression-based methods. According to the obtained results, MWCNT-TiO_2_/5W40 NF has non-Newtonian behavior. Also, the presence of NPs causes a 790% increase in μ_nf_ in the base fluid. Finally, considering R^2^ = 0.999 and a maximum error of 5%, it can be concluded that using ANN to predict the μ_nf_ of NF is acceptable. Dinesh et al. [14] investigated the influence of the φ of graphene oxide (GO) NPs on the thermophysical properties of mineral oil lubricants using ANN. The results indicate that the TC and μ_nf_ increase with increasing φ. On the other hand, these parameters have an opposite relationship and decrease with increasing Temp. In the study by Vallejo et al. [15], the maximum TC enhancement of 70% was achieved for NF with φ = 0.75 % at T = 30 °C. In this study, for the first time, mono and hybrid TiB_2_/B4C NFs based on propylene glycol: water were designed. The results indicate that mono-B4C NF has the highest thermal recovery rate (6.0 %). Also, by adding the NPs to the base fluid, the electrical conductivity improves more than 70 times. Khetib et al. [16] investigated the TC of Fe_3_O_4_/water–NF. In this study, which was done using two ANN methods along with the RSM, the TC was predicted in Fe_3_O_4_/water–NF. This study defines RSM based on several prediction functions using R-squared and MOD criteria and the ANN method based on some neurons. The results obtained from these two methods indicate that the value of R^2^ for ANN and RSM methods is 0.999 and 0.998, respectively. Also, the mean square error of the first and second methods was 0.00038 and 0.0013, respectively. ANN method has an advantage over RSM. This method can predict all points with MOD below 1%, but the RSM is only able to predict 70% of all points with MOD below 1%. In the study by Esfe et al. [17], which was carried out using the ANN, they investigated the μ_nf_ of MWCNT-MgO (25–75%)/10W40 oil HNF. The initial conditions determined in this study include the Temp range of 5–55 °C, the γ range of 6665–11997 s^−1^ and φ range of 0–1%. The most optimal method used in this study is a multilayer perceptron (MLP). The obtained results indicate that this method is highly accurate. In this study, the R^2^ values of the proposed mathematical correlation and the predicted data by ANN were estimated as 0.9321 and 0.9999, respectively. In the recent investigation conducted by Esfe et al. [18], the focus was on TC and μ_nf_ of TiO_2_/BGwater–NFs with varying compositions, notably TiO_2_/BG-water (20:80) and TiO_2_/BG-water (30:70). It is worth to mention that, RSM analysis of the TiO_2_/BG-water (20:80) NFs revealed R^2^ values of 0.9913 for TC and 0.9982 for μ_nf_. Conversely, the TiO_2_/BG-water (30:70) NFs exhibited R^2^ values of 0.9911 and 0.9993 for TC and μ_nf_ in RSM, respectively. On the other hand, the MLP model yielded R^2^ values of 0.9997 for TC and μ_nf_ in TiO_2_/BG-water (20:80) and R^2^ values of 0.999 for the same properties in TiO_2_/BG-water (30:70). Shaik et al. [19] examined the effect of synthesis conditions, encompassing Temp between 303 K and 343 K and φ ranging from 0.1% to 0.4%, on several thermophysical characteristics of M-Xene ionic fluids. Their study involved utilizing a Lowenberg-Marquardt-based ANN model and RSM for a methodical investigation of these properties, relying on experimental data. The results indicate that the optimal thermophysical properties for M-Xene IoNFs include a specific heat capacity of 2.5 J/g.K, thermal stability with weight loss of 0.33931% and μ_nf_ of 11.696 mPa s. These optimal characteristics were obtained at T= 343 K and φ=0.3% . Employing ANN, Esfe et al. [20] introduced an innovative integrated model to enhance the μ_nf_ of MWCNT-Al_2_O_3_ (40:60) hybrid nano-lubricant combined with 5W50 oil. Their study encompassed a sensitivity analysis aiming to assess the significance of various parameters governing the μ_nf_ of the MWCNT-Al_2_O_3_ (40:60)/oil 5W50 HNF , with a focus on Temp, φ, and γ within the simulation. The findings show that the highest μ_nf_ values manifest at T < 5 °C. Additionally, μ_nf_ experiences a decline with γ varying from 0 rpm to 800 rpm. Statistical analysis underscores the model's performance, demonstrating near parity with values around 0.98, 0.978, and 0.925 for the training, testing, and validation phases, respectively, with errors staying below 2.6 %. Fan et al. [21] harnessed a meticulously trained ANN via the trainlm algorithm to forecast the rheological characteristics of a water-EG/WO_3_ MWCNTs-NF. Their analysis delved into the influence of φ and Temp on the μ_nf_ of this hybrid NF. Their investigation delved into the effect of both φ and Temp on the μ_nf_ within this hybrid NF. To accomplish this, they conducted an extensive array of 42 distinct tests, incorporating seven unique φ values and six diverse Temp's to extract μ_nf_ data. The outcomes revealed the creation of a proficient ANN, trained with the trainlm algorithm, with a MSE value of 4.2e-4 and a remarkable correlation coefficient of 0.998. This demonstrates the ANN's capacity to accurately predict μ_nf_ values, offering a valuable tool for understanding and managing the NF's RB. Sahin et al. [22] investigated the stability of Fe_3_O_4_-water magnetic nanofluids (MNs) in different mass ratios using zeta potential measurements. Two ANN models were developed to predict TC and viscosity based on temperature, φ and zeta potential. The results show that these models can predict TC and viscosity using new mathematical correlations and demonstrate the potential of MNs as advanced heat transfer fluids. In a different experiment, Sahin et al. [23] predicted the zeta potential and TC of a Fe_3_O_4_/water NF using two ANNs. Three distinct network models were evaluated, and a novel mathematical correlation was suggested. High accuracy in predicting these traits was demonstrated by the findings. Despite having a larger error rate than the ANN model, the new mathematical correlation produced highly accurate thermal conductivity values calculations. Öcal et al. [24] investigated the TC of TiO_2_–CaCO_3_/water HNF at various temperatures and φ. created an ANN model and a mathematical connection to forecast thermal conductivity depending on temperature and φ. With an average error rate of 0.02% and a coefficient of determination of 0.9999, the multilayer perceptron model was chosen.

Artificial intelligence (AI) is the intelligence that a machine shows in different situations. Machine learning is a type of AI focused on building computer systems that learn from data, enabling software to improve its performance over time [[25], [26], [27], [28]]. Also, ANNs are a class of statistical learning algorithms used in machine learning and cognitive science domains [[29], [30], [31], [32], [33]]. In this study, using ANNs and different evolutionary algorithms, parameters such as μ_nf_ and TC were analyzed and estimated in silica-alumina-MWCNT/water–NF. The innovative aspect of this study lies in the utilization of ANN and various evolutionary algorithms for the analysis and estimation of parameters (μ_nf_ and TC) within the silica-alumina-MWCNT/water NFs. It introduces a fresh approach to examining the significant effect of φ and Temp on these parameters. The study showcases the novelty of the NSGA II algorithm combined with ANN and GMDH, which outperforms other algorithms and demonstrates exceptional prediction accuracy. Furthermore, the application of a GA for minimizing μ_nf_ and TC, along with the identification of optimal conditions at points A and D, represents a novel and innovative approach to enhancing NF performance.

## 2 Methodology

### 2.1 Design variables and objective functions

NFs synthesized in the laboratory and the stability of the samples is tested. The effects of temperature increase from T = 20 to T=60 °C and φ= 0.1% to φ= 0.5% on the TC and μ_nf_ of NFs are investigated. The TC is measured using the KD2-pro thermal analyzer. According to the obtained data, an experimental relationship is developed to calculate the TC. American Viscometer Brookfield model DV2 with accuracy of ± 0.1 % is used to measure the μ_nf_. This device continuously calculates and displays the viscosity of NFs at the required shear rates. After identifying the experimental data, it is necessary to extract the connection between the enter and output data. ANNs can be used to extract the relationship. The design variables in this study are φ and Temp. Also, the objective functions are μ_nf_ and TC of silica-alumina-MWCNT/water-NFs. ANNs and evolutionary algorithms will be discussed in the following. Before examining evolutionary algorithms and GMDH ANN, it is possible to examine the correlation value of the input variables and the objective functions (μ_nf_ and TC of silica-alumina-MWCNT/water–NF). If the value of this criterion is close to one or negative one, it means that there is a relationship or correlation between the two components. On the other hand, if this value is zero, it means that there is no relationship or correlation between these two components.

### 2.2 Multi-objective optimization by evolutionary algorithms

To find the best solution, mathematical optimization primarily relies on the information gleaned from the objective function's derivative. Mathematical optimizations suffer from falling into local optimal points; that is, the algorithm assumes a local optimal solution as a general and global optimal solution, and as a result, it will not be able to find a general and global optimum. Also, mathematical methods frequently cannot be used for problems whose derivative is not known or cannot be derived. Other kinds of optimization algorithms that reduce these two defects are haphazard optimizers, including meta-innovative or evolutionary methods. These methods were dependent on stochastic operators that permitted them to eschew local optimal. These methods are optimal processes. They start with making one or more accidental initial solutions to the given problem. Unlike mathematical optimization methods, stochastic methods do not need to compute the derivative of the objective function and only use the objective function to evaluate the solutions. The objective function values for the solutions are the basis for making decisions about how to enhance the solutions. Researchers used evolutionary algorithms or other methods in several studies [[34], [35], [36], [37]]. In this study, MOGOA, MALO, MOPSO, MOMFO, MOWOA and NSGA Ⅱ algorithms are used in the direction of coupling with GMDH ANN and optimization.

#### 2.2.1 MOGOA (multi-objective grasshopper optimization algorithm)

Grasshopper optimization algorithm is inspired by the life of grasshoppers. Grasshoppers belong to the insect household. They are acknowledged as pests due to the fact they cause injury to plants and crops. The living cycle of a grasshopper is depicted in Fig. 1. Although grasshoppers are typically observed in nature as a single species, they belong to one of the largest groups of all animals. The unique aspect of grasshopper swarming is that group behavior can be seen both among nymphs and among adults and adults. Nymphs in their millions leap and travel, looking like cylinder rods. When these locusts become adults, they form a group in the air and consume almost all of the vegetation they encounter on their journey. This is how locust migration occurs over large distances. The search process is logically divided into two parts by algorithms based on nature: exploration and exploitation. During the exploration phase, search agents are encouraged to move at random, whereas, during the exploitation phase, they typically move locally and around their location. These two actions, as well as the search for the target, are performed naturally by the locust. Therefore, it has been tried to find a method for mathematical modeling of this behavior, which is referred to later on its mathematical characteristics [38]. Eq. (1) [39] was the initial calculation for the mathematical model:

(1) $$X_{i}=S_{i}+G_{i}+A_{i}$$

where $A_{i}$ depicts the grasshopper's direction, $X_{i}$ the position of the grasshopper, $S_{i}$ the social interaction, and G, the gravity force applied to the grasshopper. The value of S_i_, which means social interaction for the i-th locust, is calculated according to Eq. (2) [38]:

(2) $$S_{i}=\sum_{j=1}^{N}s\left(d_{\text{ij}}\right)\hat{d_{\text{ij}}}$$

where the expression represents the distance between the i-th and j-th propellers $d_{\text{ij}}$ and is calculated as Eq. (3) [38]:

(3) $$d_{\text{ij}}=\left|x_{i}-x_{j}\right|$$

**Fig. 1:** Correlation value between input variables and objective functions.

As shown in Eq.2, S is a function that defines the pressure of social force; the unit vector $d_{\text{ij}}$ connects the i-th locust to the j-th locust. Eq. (4) [38] is the formula used to calculate the social force's function S:

(4) $$S\left(r\right)=fe^{\frac{-r}{I}}-e^{-r}$$

Where I denote the length of the gravity scale and f denotes the gravity's intensity. Research has shown that Eq. (1) [39] cannot be used in crowd simulation and optimization algorithms because this relationship hinders exploration and exploitation in the search area round a solution. In point of fact, the model has been applied to crowding in open space. As a result, Eq. (5) [38] is utilized, which is capable of simulating the swarm's interaction between locusts.

(5) $${x_{i}}^{d}=c\left({\sum_{j=1}^{N}c\frac{Ub_{d}-lb_{d}}{2}s\left({x_{j}}^{d}-{x_{i}}^{d}\right)\frac{x_{j}-x_{i}}{d_{\text{ij}}}}_{j\neq i}\right)+\hat{T_{d}}$$

In this equation, S is obtained from Eq. (4) [38], and the gravity parameter (G) is the wind direction (A) it is not considered. In Eq. (5) [38], the adaptive parameter c is used twice for the following reasons:

• The prime c from the left is very analogous to the internal weight (W) in the PSO algorithm. It decreases the motions of the propellers round the target.
• The second variable c reduces the area of attraction, repulsion and tranquility between the propellers. Consider the component $c\frac{Ub_{d}-lb_{d}}{2}s\left({x_{j}}^{d}-{x_{i}}^{d}\right)$, where $\frac{Ub_{d}-lb_{d}}{2}$ it linearly reduces the space between the propellers that have to perform exploration and exploitation.

In short, the first part of Eq. (1) [39] and 2 [38] considers the position of other locusts and simulates the transaction between the locusts in nature, and the second part, i.e., $\hat{T_{d}}$, simulates the tendency of the locusts to movement to the food source. Also, the c parameter simulates the decrease in the speed of the locusts when they approach the food source and finally eat it. The search space can be explored and exploited using the proposed mathematical formula. The level of exploration and exploitation of search agents must, however, be adjusted via a mechanism. Because they do not have wings during the larval stage, grasshoppers first move around and look for local food in the natural world. After that, they explore a larger area while moving freely through the air. Exploration, on the other hand, takes precedence in random optimization algorithms due to the requirement to locate search space regions with greater potential. The exploitation requires the search agents to look locally for a good match to the global optimum after discovering more promising areas. To maintain the balance between exploration and exploitation, the parameter c needs to decrease with increasing iteration times and during the algorithm. The coefficient c reduces the comfort zone in proportion to the number of repetitions, shown in Eq. (6) [38] how to calculate it.

(6) $$C=C_{\max}-i\frac{c_{\max}-c_{\min}}{l}$$

Where C_max_ is the highest value, C_min_ is the lowest value, and i shows the current iteration number and the maximum number of times the algorithm is repeated.

The grasshopper optimization algorithm consists of the following steps.

1. In the search area, a population of locusts is created at random.
2. Determining the value of the parameters of the problem, including the lower bound (C_min_) and upper bound (C_max_) of the comfort zone and the maximum number of development cycles.
3. Calculate the fitness of each propeller using the optimization function
4. Identifying the ideal grasshopper (grasshopper with better fitness) in variable T
5. As long as the termination condition is not reached (I < maximum of iteration)
  • Updating the comfort zone by Eq. (6) [38].
  • For each grasshopper:
  • The distances between grasshoppers are normalized in Refs. [[40], [41]] in each iteration
  • Using Eq. (5) [38], update each grasshopper's location.
  • A grasshopper that has left the search space should be brought back to it.
  • T will be updated if a grasshopper with a better fit is found.
  • Adding the internal iteration number of the algorithm (l = l+1)
6. Returning the best grasshopper as the final answer.

#### 2.2.2 MALO (multi-objective Ant lion optimization algorithm)

The ant lion worm is often called the "hole burrowing bug" because it digs holes in the sand while searching for a good position to set up a trap [42]. During the hunting process, the ant lion creates holes in the soft and sandy ground and then waits patiently at the bottom of the hole. When the prey slips into the hole, it is immediately hunted by the ant lion. Or, if the prey is trying to escape, the ant lion starts sprinkling sand grains on the edges of the hole to make the prey slide to the bottom of the hole. When the caterpillar of the ant worm sprinkles the sand from the bottom of the hole to the sides, it causes the edges to fall, which causes the prey to fall and guides it toward the hunter. The optimal adaptation algorithm of the anthill is a new meta-heuristic algorithm that is inspired by the nature and the hunting mechanism of the interaction between the anthill and the ant [42]. This algorithm uses the reaction between the anthill and the trapped ants. The anthill optimizer has very good results in terms of exploration. It provides improved, local optimal avoidance, exploitation and convergence [42]. The main advantage of the ant lion optimizer algorithm is its high convergence rate and utilization. The main reason for this speed of convergence and high exploitation is the mechanism of margin reduction and comparative elitism. Conversely, the high utilization of the ant lion optimization algorithm is due to the use of rotating turn selection mechanisms and random walking, which provides the possibility of population diversity. In the primary reference for the anthill optimization algorithm [42], we first consider the ant to be movable in the search space before permitting the anthill to hunt it To model its behavior. This movement is modeled using Eq. (7) [42] because the ant moves randomly around the area:

(7) $$X\left(t\right)=\left[0,\mathrm{cumsum}\left(2r\left(t_{1}\right)-1\right),\mathrm{cumsum}\left(2r\left(t_{2}\right)-1\right),\ldots ,\mathrm{cumsum}\left(2r\left(t_{n}\right)-1\right)\right]$$

In Eq. (7) [42], cumsum calculates the cumulative sum, n represents the most repetition, t is the expression of the phase of the random walk (t-th repetition in this time), (r(t) is an accidental function that takes the form of Eq. (8) [42].

(8) $$r\left(t\right)=\left\{ \begin{array}{c} 1\;\mathrm{if}\;\mathrm{rand}>0.5\\ 0\;\mathrm{if}\;rand\leq 0.5 \end{array}\right.$$

In Eq. (8) [42], t represents the stage of random walk, and r is a random number in the interval [0,1]. The position of ants is stored in the matrix of Eq. (9) [42] and used during optimization.

(9) $$M_{\text{Ant}}=\left[\begin{array}{ccccc} A_{1,1} & A_{1,2} & \cdots & \cdots & A_{1,d}\\ A_{2,1} & A_{2,2} & \cdots & \cdots & A_{2,d}\\ \cdots & \cdots & \cdots & \cdots & \cdots \\ \cdots & \cdots & \cdots & \cdots & \cdots \\ A_{n,1} & A_{n,2} & \cdots & \cdots & A_{n,d} \end{array}\right]$$

In Eq. (9) [42], $M_{\text{Ant}}$ determines the position of every ant, $A_{i,j}$ specifies the j-th variable of the i-th ant. n specifies the number of ants, and d specifies the number of variables. During optimization, a fitness function is utilized to evaluate each ant. After that, these functions are saved as Eq. (10) [42].

(10) $$M_{\text{OA}}=\left[\begin{array}{c} f\left(A_{1,1}\;A_{1,2\;}\cdots \cdots A_{1,d}\right)\\ f\left(A_{2,1}\;A_{2,2\;}\cdots \cdots A_{2,d}\right)\\ \cdots \cdots \cdots \cdots \cdots \\ \cdots \cdots \cdots \cdots \cdots \\ f\left(A_{n,1}\;A_{n,2\;}\cdots \cdots A_{n,d}\right) \end{array}\right]$$

This matrix stores the value of each ant's fitness function in the ant lion optimization algorithm. It is expected that the subterranean insects are concealed in a space. Matrices of Equations are used to store this position and its objective function. Uses include Eq. (11) [42] and Eq. (12) [42].

(11) $$M_{\text{Antlion}}=\left[\begin{array}{ccccc} {\text{AL}}_{1,1} & {\text{AL}}_{1,2} & \cdots & \cdots & {\text{AL}}_{1,d}\\ {\text{AL}}_{2,1} & {\text{AL}}_{2,2} & \cdots & \cdots & {\text{AL}}_{2,d}\\ \cdots & \cdots & \cdots & \cdots & \cdots \\ \cdots & \cdots & \cdots & \cdots & \cdots \\ {\text{AL}}_{n,1} & {\text{AL}}_{n,2} & \cdots & \cdots & {\text{AL}}_{n,d} \end{array}\right]$$

(12) $$M_{\text{OAL}}=\left[\begin{array}{c} f\left({\text{AL}}_{1,1}\;{\text{AL}}_{1,2\;}\cdots \cdots {\text{AL}}_{1,d}\right)\\ f\left({\text{AL}}_{2,1}\;{\text{AL}}_{2,2\;}\cdots \cdots A_{L2,d}\right)\\ \cdots \cdots \cdots \cdots \cdots \\ \cdots \cdots \cdots \cdots \cdots \\ f\left({\text{AL}}_{n,1}\;{\text{AL}}_{n,2\;}\cdots \cdots {\text{AL}}_{n,d}\right) \end{array}\right]$$

In Eq. (11) [42] and Eq. (12) [42], $M_{\text{Antlion}}$ and $M_{\text{OAL}}$ define the position matrix and objective function matrix of each ant lion, respectively. During the optimization, the following steps are applied.

• Ants move randomly throughout the search space.
• Random walk is applied to all dimensions of ants.
• Random walking is affected by the ant trap.
• Ants can dig bigger pits according to their objective function (the bigger the objective function, the bigger the pit is)
• With a bigger pit, the ant lion can take more ants.
• An anthill can hunt every ant.
• The ant reduces its walking range in response to the ant lion traps.
• When an ant lion hunts an ant, it means that the ant is taken captive and dragged beneath the sand.
• To catch the next ant, the anteater moves around after each hunt and builds a pit with the right changes.

The accidental motion of ants is based on Eq. (7) [42]. In every step of optimization, ants update their position with random walking. For ants to walk randomly in the search space, they are normalized by Eq. (13) [42].

(13) $${X_{i}}^{t}=\frac{\left({X_{i}}^{t}-a_{i}\right)\times \left(d_{i}-{c_{i}}^{t}\right)}{\left({d_{i}}^{t}-a_{i}\right)}$$

Here, a_i_ is the minimum random walk at the i-th position; d_i_ is the maximum random walk at the i-th position; C_i_^t^ is the minimum i-th variable in the t-th iteration, and tid is the maximum i-th variable in the t-th iteration. To express it mathematically, Eq. (14) [42] and 15 [42] are expressed.

(14) $${c_{i}}^{t}={{\text{Antlion}}_{j}}^{t}+c^{t}$$

(15) $${d_{i}}^{t}={{\text{Antlion}}_{j}}^{t}+d^{t}$$

The value of all variables in the t-th iteration is represented by the minimum of C^t^ in Eq. (14) [42] and Eq. (15) [42], while the value of the vector containing the maximum of all variables in the t-th iteration is represented by d^t^. Also, C_i_^t^ is the lowest value of all the variables in the -ith ant and d_it is the vector with the highest value. In this regard, ${{Antlion}_{j}}^{t}$ represents the j-th position of the ant lion in the t-th iteration. To model the hunting ability of ants, the roulette wheel structure is used. The anthill optimization algorithm needs a rotating wheel operator to determine the anthills based on their fitness function during the optimization. When an ant is caught in the trap, the anthill throws stones toward the edges of the pit, and its mathematical model is in the form of Eq. (16) [42] and 17 [42] is defined.

(16) $$c^{t}=\frac{c^{t}}{I}$$

(17) $$d^{t}=\frac{d^{t}}{I}$$

In Eq. (16) [42] and 17 [42], I is a fixed and minimum ratio of all variables in the t-th repetition, including the vector with the maximum value of the variables in the t-th repetition. I is defined as Eq. (18) [42].

(18) $$I=10^{w}\frac{t}{T}$$

In Eq. (18) [42], where t is the current number of repetitions, T is the maximum number of repetitions, and w is a constant that is defined as Eq. (19) [42] based on the current number of repetitions.

(19) $$w=\left\{ \begin{array}{c} 2\;\mathrm{when}\;t>0.1T\\ 3\;\mathrm{when}\;t>0.5T\\ 4\;\mathrm{when}\;t>0.75T\\ 5\;\mathrm{when}\;t>0.9T\\ 6\;\mathrm{when}\;t>0.95T \end{array}\right.$$

When the prey reaches the bottom of the trap and is placed in the ant lion's mouth, the final stage of hunting has occurred. The milk ant eats the prey by dragging it into the sand after this stage. When this method is used, it is assumed that the ant is hunting when it is buried in the sand. The position of the anthill should then be updated in comparison to the position from which the ant was hunted to increase the likelihood of a new hunt. Eq. (20) [42] demonstrates this act.

(20) $${{\text{Antlion}}_{j}}^{t}={{\text{Ant}}_{j}}^{t}\;\mathrm{if}\;f\left({{\text{Ant}}_{i}}^{t}\right)>f\left({{\text{Antlion}}_{i}}^{t}\right)$$

In Eq. (20) [42], t indicates the execution repetition number and ${{Antlion}_{j}}^{t}$ indicates the position of the j-th ant in the tth repetition and indicates the position of the i-th ant in the t-th repetition.

#### 2.2.3 MOMFO (multi-objective Moth flame optimization algorithm)

In nature, the type of movement of butterflies is in transverse orientation, which is the main idea of this optimization method. This algorithm [43] was compared with other prominent algorithms inspired by nature in 29 criterion functions and 7 actual engineering problems. These functions' statistical results demonstrate that this algorithm is capable of producing precise and competitive outcomes. What's more, the aftereffects of genuine issues show the upsides of this calculation in tackling testing issues with restricted and obscure hunt spaces. The unique way that butterflies navigate at night is an intriguing fact. They use a horizontal orientation mechanism for guidance as they fly at night under the moonlight. A butterfly flies in this manner by maintaining a constant angle to the moon, which is an extremely efficient method for traveling long distances in a straight line [44,45]. The butterflies are assumed to be potential solutions in this algorithm, and their locations in space serve as the problem's variables. Therefore, butterflies can move in a one-dimensional, two-dimensional, or multi-dimensional space. Since the flame-propeller optimization algorithm is a population-based algorithm, the set of propellers is a matrix of n×d order. Eq. (21) [43] gives the matrix of the propeller set.

(21) $$M=\left[\begin{array}{ccccc} M_{1,1} & M_{1,2} & \cdots & \cdots & M_{1,d}\\ M_{2,1} & M_{2,2} & \cdots & \cdots & M_{2,d}\\ \cdots & \cdots & \cdots & \cdots & \cdots \\ \cdots & \cdots & \cdots & \cdots & \cdots \\ M_{n,1} & M_{n,2} & \cdots & \cdots & M_{n,d} \end{array}\right]$$

In Eq. (21) [43], n is the number of butterflies, and d is the number of variables or the number of dimensions of the search space for the optimal solution. Also, in this algorithm, an n vector is defined for the usefulness of butterflies. Eq. (22) [43] shows the utility vector of butterflies. In Eq. (22) [43], where n is the total number of butterflies and ${OM}_{i}$ is the utility function value for the i-th butterfly.

(22) $$\text{OM}=\left[\begin{array}{c} {OM}_{1}\\ {OM}_{2}\\ \vdots \\ {OM}_{n} \end{array}\right]$$

Another key concept in the flame-propeller optimization algorithm is flames. The set of flames is also like the set of the propeller in the form of an n×d matrix. Eq. (23) [43] shows the matrix of the set of flames.

(23) $$F=\left[\begin{array}{ccccc} F_{1,1} & F_{1,2} & \cdots & \cdots & F_{1,d}\\ F_{2,1} & F_{2,2} & \cdots & \cdots & F_{2,d}\\ \cdots & \cdots & \cdots & \cdots & \cdots \\ \cdots & \cdots & \cdots & \cdots & \cdots \\ F_{n,1} & F_{n,2} & \cdots & \cdots & F_{n,d} \end{array}\right]$$

In Eq. (23) [43], where n represents the number of flames and d represents the number of variables or dimensions of the search space for the best answer. Also, in this algorithm, an n vector is defined for the utility of the flames. Eq. (24) [43] shows the utility of the flames. In Eq. (24) [43], n is the number of flames, and OF shows the utility function value of the i-th flame.

(24) $$\mathrm{OF}=\left[\begin{array}{c} {\text{OF}}_{1}\\ {\text{OF}}_{2}\\ \vdots \\ {\text{OF}}_{n} \end{array}\right]$$

It is important to note that flames and butterflies are both potential neighbors. The only thing that separates them is how they act and how to update them. Butterflies are real search agents that search the problem-solving space, while flames are the best butterflies ever obtained. In this algorithm, each butterfly moves around a flame, and when a candidate solution finds a better one, it will update the new candidate's answer with the latest flame. A butterfly never fails to find the best solution, thanks to this mechanism. The flame-butterfly optimization algorithm is a triad that, for solving optimization problems, roughly identifies the global optimal solution. Eq. (25) [43] gives the mathematical model of the flame-propeller optimization algorithm.

(25) MFO=(I,P,T)

In Eq. (25) [43], I is a function that randomly selects a set of primary candidate answers. This set of answers is considered a set of butterflies. The scientific model of function I is defined in Eq. (26) [43].

(26) I;∅→{M,OM}

The algorithm's primary function is the P function. This function moves butterflies in the search space. In each step, this function receives a matrix M and updates the location of the propellers in that matrix. Then, it returns the updated matrix M. The scientific model of P function is shown in Eq. (27) [43].

(27) P:M→M

The algorithm's end criterion is examined by the T function. If the end criterion is satisfied, it returns true. Otherwise, it returns false. Eq. (28) [43] depicts the scientific model of the T function.

(28) T:M→{true,false}

Additionally, this algorithm defines 2 d vectors, lb and ub, that represent the propellers' respective lower and upper limits. Eq.s (29) [43] and 30 [43] depict the vectors lb and ub, where ${\text{lb}}_{i}$ and ${\text{ub}}_{i}$ represent the lower and upper limits on the propeller's i-th position, respectively.

(29) $$\mathrm{lb}=\left\{{\text{lb}}_{1},{\text{lb}}_{2},\cdots ,{\text{lb}}_{d}\right\}$$

(30) $$\mathrm{ub}=\left\{{\text{ub}}_{1},{\text{ub}}_{2},\cdots ,{\text{ub}}_{d}\right\}$$

As mentioned before, the flame-propeller algorithm uses the behavior of the propeller concerning the flame, called transverse direction. Eq. (31) [43] shows the mathematical model of the behavior of the propeller, in which the $M_{i}$ propeller updates its location according to the j-th flame. The S function also creates a spiral motion for the propeller. Any spiral function can be used in this algorithm. Eq. (32) [43] shows the proposed spiral function.

(31) $$M_{i}=S\left(M_{i},F_{j}\right)$$

(32) $$S\left(M_{i},F_{j}\right)=D_{i}.e^{\text{bt}}.\cos\left(2\pi t\right)+F_{j}$$

In Eq. (32) [43], the Euclidean term $D_{i}$ is the i-th propeller of the j-th flame, and b is a constant number to create a spiral movement. In this research, b = 1 is considered. t is also a random number in the closed interval [−1,1]. Eq. (33) [43] and 34 [43] get a random number in the interval t.

(33) $$a=-1-\frac{\text{Iteration}}{\mathrm{Maximum}\;\mathrm{Iteration}}$$

(34) t=((a−1)*rand)+1

Eq. (35) [43] shows the Euclidean distance between the middle of the butterfly and the middle of the flame.

(35) $$D\left(i,j\right)=\left|M_{i,j}-F_{i,j}\right|$$

The main part of the flame-propeller optimization algorithm is the helical motion of the propeller around the flame. However, if the number of flames is equal to the size of the propellers, the time of the process of extracting the optimal solution increases. For this purpose, an adaptive mechanism is provided in this algorithm to reduce the number of flames. In each step, as many as flame_no from the sorted set of butterflies are considered as a set of flames. Eq. (36) [43] obtains the value of flame_no in each step.

(36) $$flame\_no=\mathrm{round}\left(N-l*\frac{N-1}{T}\right)$$

Eq. (36) [43] shows the number of flames in each stage of the algorithm execution. L and T, respectively, show the number of recent execution stages and the maximum execution stage of the flame-propeller optimization algorithm. N also shows the maximum number of flames. The P function is executed iteratively following the initial initialization until the T function returns the termination condition.

#### 2.2.4 NSGA II (non-dominated sorting genetic algorithm)

In addition to all the applications of the meta-heuristic genetic algorithm with non-dominant sorting, it can be called the template for the formation of most multi-objective optimization algorithms. The binary tournament selection function is used to select a few of the answers from each generation for the problem in the meta-heuristic genetics algorithm with non-dominant sorting [46].In the binary selection function, two answers to the problem are chosen at random from the population, then they are compared, and the superior answer is chosen in the end. The rank of the answer to the problem and the density distance related to the answer to the problem are the selection criteria in the meta-heuristic genetic algorithm with non-dominated sorting. The lower the position worth of the response for the issue and the more noteworthy the pressure distance for the issue, the more helpful it is. Each generation's sets of answers are chosen to participate in crossover and mutation by repeating the binary selection function on the population. The operation of intersection is carried out on a portion of the set of selected answers, and the operation of mutation is carried out on the remaining ones, resulting in the production of a population of children and mutants. This population and the initial population are combined in the sequence. The newly formed population is initially sorted in ascending order by rank. Members of the population who have the same rank are sorted according to the density distance criterion and in descending order. The answers are then selected from the top of the sorted list, equal to the number of answers from the main population, and the remaining members of the population are discarded. The next generation is made up of the selected members of the population, and the cycle described in this section is repeated until the algorithm's termination conditions are met. The non-dominated solutions obtained from solving the meta-heuristic genetic algorithm with non-dominated sorting for the problem are often known as the Pareto front. In the meta-heuristic genetic algorithm with non-dominated sorting, none of the Pareto front solutions will be preferred over the others. And each of them might be the best option for resolving the issue, depending on the circumstances. In the following, the steps of the genetic meta-heuristic algorithm with non-dominated sorting for the problem have been examined.

1. Generate an initial random population. $P_{0}$ of size N, set value t = 0.
2. Combination and mutation functions should be applied on $P_{0}$ to produce a population of children of $Q_{0}$ with size N.
3. If the termination condition is met, the algorithm is stopped and $P_{t}$ is returned.
4. Put$R=P_{t}\cup Q_{t}$
5. The meta-heuristic genetic algorithm with non-dominant sorting should be used to detect the non-dominant fronts. $F_{1},...,F_{k}$ in $R_{t}$.
6. For i=1,2,3,...,k, perform the following steps:
  • The crowding distance criterion of the answers should be extracted in the *Fi* front.
  • The population of answers $P_{t+1}$ should be created as follows:
    ⁃ If $|P_{t+1}\left|+\right|F_{i}|\leq N$, so $P_{t+1}=P_{t+1}\cup F_{i}$.
    ⁃ If $|P_{t+1}\left|+\right|F_{i}|\;>\;N$, so the number of $N\;-\;|P_{t+1}|\;$ Add $P_{t+1}$ from the answers with the lowest congestion distance values.
7. Select parents from $P_{t+1}$ by using the binary selection function based on the crowding distance criterion. Apply combination and mutation functions on $P_{t+1}$ to create a population of $Q_{t+1}$ with size N.
8. Set the value of t = t+1 and go to step 3.

#### 2.2.5 MOPSO (multi-objective particle swarm optimization)

The MOPSO algorithm is a special case of the PSO algorithm [47]. The PSO algorithm is a social search algorithm that is modeled on the social behavior of flocks of birds. In PSO, particles flow in the search space. The basis of PSO work is based on the principle that at any moment, each particle adjusts its location in the search space according to the best location it has been in so far and the best location in its entire neighborhood. Many real-world problems have two or more goals. In these problems, goals may conflict with each other and reach the optimal point with an interaction between possible solutions. The PSO algorithm is a unified single-objective optimizer, while in multi-objective problems, there is often no optimal global optimal point. Therefore, To create a PSO algorithm capable of solving multi-objective optimization problems, some modifications are needed. The individual best performance of each particle ($p_{\text{best}}$) is replaced by the new answer if and only if it leads to a better $p_{\text{best}}$ formation. Also, in the process of updating the global best performance ($g_{\text{best}}$), two important issues should be considered.

• Proper allocation and selection must be done so that a search can move toward the set of Pareto optimal points;
• The diversity of particles should be maintained to prevent an early convergence and obtain optimal distributed Pareto points.

The PSO method is an optimization technique based on probability rules that use the social behavior of birds while searching for food to guide the population to the promising region in the search space, which is suitable for solving complex problems and has a considerable speed. Eberhart and Kennedy proposed this approach as an alternative to the genetic algorithm. Due to its advantages over other optimization techniques, this method has been used a lot in recent years. One of the benefits is that this technique doesn't have to ascertain subordinates. So that the information related to the appropriate solution is kept in all the components and the components share the information. It can also be used for random objective functions because it is less sensitive to the objective function itself. PSO is simple to program, requires fewer parameters to be combined, and the optimal value can be determined independently of the initial solution. Particles are the solution method in PSO, and their movement throughout the search space is determined by the new group's instructions. Eq. (37) [47] and 38 [47] govern how the primary PSO algorithm operates to determine the particle's subsequent location:

(37) $$V_{i+1}\left(j\right)=V_{i}\left(j\right)+c_{1}.r_{1,i}\left(j\right).\left(p_{\text{best}}\left(j\right)-x_{i}\left(j\right)\right)+c_{2}.r_{2,i}\left(j\right).\left(g_{\text{best}}\left(j\right)-X_{i}\left(j\right)\right)$$

(38) $$X_{i+1}\left(j\right)=V_{i+1}\left(j\right)+X_{i}\left(j\right)$$

i is the number of repetitions, and j is the optimization vector variable. $X_{i}\left(j\right)$ is the value of variable j in the i-th repetition, and $V_{i}\left(j\right)$ is equal to the speed of the variable j in the i-th repetition. $r_{1,i}$, $r_{2,i}$ are random variables that are in the range [1and0] $p_{\text{best}}\left(j\right)$ is equal to the value of variable j obtained from the best solution of the special particle up to i-th iteration, and $g_{\text{best}}\left(j\right)$ is equal to the value of variable j obtained from the best collective solution. The speed of each particle should be in the range $\left[-V_{\max},V_{\max}\right]$ to reduce the probability of the particle leaving the problem space. To balance between detection and extraction in the PSO algorithm, it is suggested to use algebraic weight (w) according to Eq. (39) [47]:

(39) $$V_{i+1}\left(j\right)=w.V_{i}\left(j\right)+c_{1}.r_{1,i}\left(j\right).\left(p_{\text{best}}\left(j\right)-x_{i}\left(j\right)\right)+c_{2}.r_{2,i}\left(j\right).\left(g_{\text{best}}\left(j\right)-X_{i}\left(j\right)\right)$$

During the optimization iterations, the value of w decreases linearly to 0.4 from the initial value of 0.9.

#### 2.2.6 MOWOA (multi-objective whale optimization algorithm)

This algorithm was presented by Mirjalili and Lewis [48]. By using the collective intelligence of particles, this algorithm can find the best paths to the source. While this problem does not exist in other meta-engineering algorithms, and other algorithms focus more on optimizing a system, this algorithm is intrinsically suitable for problems Routing is designed. The favorite prey of whales is small fishes. The unique method of hunting that whales use is truly remarkable. The bubble feeding method is the name given to this behavior. These whales tend to feed small fish near the surface of the H_2_O. It was estimated that This style of hunting is done by creating bubbles along a circle or paths. The Wall algorithm is one of the optimization algorithms that is inspired by nature and is used in various fields. To find the optimal solution, the whales try to make the following three important movements around the current optimal solution, which is also assumed to be the location of the fish shoal, which can be seen in Fig. 4(a–c).

• Spiraling up
• Double round
• Random movement

They are surrounded by whales after locating the hunting area. The WOA algorithm assumes that the hunting target or a close match to the optimal state is the current best-candidate solution because the optimal design location in the search space is unknown. Other search agents attempt to update their location with the best search agent after the best agent Search is identified. Eq. (40) [48] and 41 [48] are used to express this behavior.

(40) $$D=\left|\vec{C}\;.\;\vec{X^{*}}\left(t\right)-\vec{X}\left(t\right)\right|$$

(41) $$\vec{X}\left(t+1\right)=\vec{X^{*}}\left(t\right)-\vec{A}\;.\;\vec{D}$$

where t is the current iteration, A and C are the coefficient vectors, $X^{*}$ is the position vector of the best solution so far, and X is the object's location vector. It should be noted that every iteration of this process necessitates updating. $X^{*}$ and selecting the best solution. Eq. (42) [48] is used to calculate vectors A and C:

(42) $$\vec{A}=2\vec{a}.\vec{r}-\vec{a},\vec{C}=2\vec{r}$$

During the iteration period (in both the exploration and exploitation phases), $\vec{a}$ is a linear vector that has been reduced from 0 to 2. Additionally, $\vec{r}$ is a random vector in the [0,1] range. As seen in Fig. 7, the first approach to calculate the distance between whales located in |X,Y| and the prey located at $\left(X^{*},Y^{*}\right)$ is a spiral equation created between the position of the whale and the prey. The imitation of the humpback whale's spiral motion is given in Eq. (43) [48]:

(43) $$\vec{X}\left(t+1\right)=\vec{\overset{´}{D}}e^{\text{bl}}.\;\cos\left(2l\right)+\vec{X^{*}}\left(t\right)$$

It is important to keep in mind that the humpback whale swims in a spiral and a circular pattern around its prey. Eq. (44) [48] describes the mathematical model as follows:

(44) $$\vec{X}\left(t+1\right)=\left\{\begin{array}{c} \vec{X^{*}}\left(t\right)-\vec{A}\;.\;\vec{D}\;\mathrm{if}\;p<0.5\\ \vec{\overset{´}{D}}e^{\text{bl}}.\;\cos\left(2l\right)+\vec{X^{*}}\left(t\right)\;\mathrm{if}\;p>0.5 \end{array}\right\}$$

In contrast to the exploitation phase, the position of a search agent in the exploration phase is selected instead of the best search agent and is randomly updated based on the search agent. The mathematical model is as described in Eq. (45) [48] and 46 [48]:

(45) $$D=\left|\vec{C}\;.\;\vec{X_{\text{rand}}}-\vec{X}\right|$$

(46) $$\vec{X}\left(t+1\right)=\vec{X_{\text{rand}}}-\vec{A}\;.\;\vec{D}$$

A random position vector is $\vec{X_{\text{rand}}}$. Search agents select and update their positions at random during each iteration based on which search agent found the best solution.

### 2.3 ANNs (group method of data handling (GMDH))

ANNs are utilized in diverse problems, including regression , classification [49,50], patternization [51], time series prediction [35] and clustering [52,53]. For forecasting a mathematical relationship from the simulated data, a regression operation should be conducted. In this study, GMDH ANN is used to perform regression operations. This ANN type has been employed by researchers in diverse fields of engineering [,^35^,[54], [55], [56], [57], [58]]. The production and prediction of meaningful output data is the primary objective of GMDH ANN. The input layer, the hidden layer, and the output layer are the three general layers that make up this ANN. Each neuron carries a polynomial equation because the inputs are gathered in the form of $\left(\begin{array}{c} n\\ 2 \end{array}\right)$ combinations. The neurons are combined similarly to reach the final layer, also known as the output layer. The input function and the output value of the GMDH ANN are, respectively, x and y. The approximate function of f is the estimated output value that is predicted by ANN with $\hat{y}$ and also $\hat{\;f}$. In functions with multiple inputs M and one output n, the actual values are determined using Eq. (47) [59].

(47) $$y=f\left(x_{i1},x_{i2},x_{i3},\ldots .,x_{\text{in}}\right)\left(\;i=1,2,3,\ldots ,M\right)$$

The values of $\hat{y}$ are predicted by the function $\hat{\;f}$ with the input vector of $X=\left(x_{i1},x_{i2},x_{i3},\ldots .,x_{\text{in}}\right)$ and its equation is tested according to Eq. (48) [59].

(48) $${\hat{y}}_{i}=\hat{f}\left(x_{i1},x_{i2},x_{i3},\ldots .,x_{\text{in}}\right)\left(\;i=1,2,3,\ldots ,M\right)$$

The error squared value that must be minimized between the output and the output that is approximated by GMDH must be calculated in the subsequent step. The least squared error equation between these two outputs is estimated based on Eq. (49) [59].

(49) $$\sum_{i=1}^{M}{\left[\hat{f}\left(x_{i1},x_{i2},x_{i3},\ldots .,x_{\text{in}}\right)-{\hat{y}}_{i}\right]}^{2}\;\to \;\min$$

The Volterra series connects the inputs and outputs [60], whose relationship is according to Eq. (50) [60].

(50) $$y=a_{0}+\sum_{i=1}^{n}a_{i}x_{i}+\sum_{i=1}^{n}\sum_{j=1}^{n}a_{\text{ij}}x_{i}x_{j}+\sum_{i=1}^{n}\sum_{j=1}^{n}\sum_{k=1}^{n}a_{\text{ijk}}x_{i}x_{j}x_{k+}\ldots \text{.}$$

The polynomials analyzed in Eq. (50) [60] are arranged as Eq. (51) [59] by the Kolmogorov-Gabor polynomials.

(51) $$\hat{y}=G\left(x_{i},x_{j}\right)=a_{0}+a_{1}x_{i}+a_{2}x_{j}+a_{3}{x_{i}}^{2}+a_{4}{x_{j}}^{2}+a_{5}x_{i}x_{j}$$

The $a_{i}$ coefficients are determined using regression, and Eq. (47) [59] and 48 [59] are explained by Eq. (52), which must be minimized.

(52) $$E=\frac{\sum_{i}^{M}{\left(y_{i}-G_{i}\right)}^{2}}{M}\;⟶\min$$

Using least square error logic and polynomial regression in Eq. (48), the best outputs can be anticipated. To evaluate the performance of GMDH ANN with evolutionary algorithms, they should be evaluated with criteria. To evaluate the performance of GMDH ANN with evolutionary algorithms, they should be evaluated with criteria. In this study, 6 measures of RMSE, R, MSE, R^2^, MAPE and MAE are used. These criteria are discussed in the form of Eqs. (53), (54), (55), (56), (57), (58)).

(53) $$R=\frac{\sum_{i=1}^{n}\left(y_{i,\mathrm{Experiment}}-{\bar{y}}_{i,\mathrm{Experiment}}\right)\left(y_{i,\mathrm{ANN}}-{\bar{y}}_{i,\mathrm{ANN}}\right)}{\sqrt{\sum_{i=1}^{n}{\left(y_{i,\mathrm{Experiment}}-{\bar{y}}_{i,\mathrm{Experiment}}\right)}^{2}\sum_{i=1}^{n}{\left(y_{i,\mathrm{ANN}}-{\bar{y}}_{i,\mathrm{ANN}}\right)}^{2}}}$$

(54) $$\mathrm{RMSE}=\sqrt{\frac{\sum_{i=1}^{n}{\left(y_{i,\mathrm{ANN}}-y_{i,\mathrm{Experiment}}\right)}^{2}}{n}}$$

(55) $$\mathrm{MAE}=\frac{\sum_{i=1}^{n}\left|y_{i,\mathrm{ANN}}-y_{i,\mathrm{Experiment}}\right|}{n}$$

(56) $$\mathrm{MSE}=\frac{\sum_{i=1}^{n}{\left(y_{i,\mathrm{ANN}}-y_{i,\mathrm{Experiment}}\right)}^{2}}{n}$$

(57) $$R^{2}=1-\sum_{i=1}^{n}\frac{{\left(y_{i,\mathrm{ANN}}-y_{i,\mathrm{Experiment}}\right)}^{2}}{{y_{i,\mathrm{Experiment}}}^{2}}\;$$

(58) $$\mathrm{MAPE}=\frac{\sum_{i=1}^{n}\left|\frac{y_{i,\mathrm{ANN}}-y_{i,\mathrm{Experiment}}}{y_{i,\mathrm{Experiment}}}\right|}{n}\times 100$$

Deviation analysis of the μ_nf_ ratio was used to determine this correlation's (R) accuracy. Eq. (59) can be used to calculate the difference between the results predicted by the correlation and those found in the experiments []:

(59) $$\mathrm{MOD}=\left(\frac{{Objective\;function}_{\mathrm{Exp}}-{Objective\;function}_{\text{ANN}}}{{Objective\;function}_{\mathrm{Exp}}}\right)\times 100$$

The data is divided in such a way that 70% of the data is considered for training data and the rest of the data is considered for testing data. The GMDH algorithm, like other machine learning algorithms, has a prediction function known as Kolmogorov-Gabor whose equation is according to Eq. (51). To obtain the optimal prediction points, the GMDH approach should be applied in combination with evolutionary optimization techniques. For this, the number of neurons, the number of hidden layers, and the pressure coefficient have all been selected as optimization technique variables. The number of neurons in the hidden layer is considered to be one as the composition $\left(\begin{array}{c} n\\ 2 \end{array}\right)$ states that there can only be one neuron in each layer. It is believed that the number of hidden layers ranges from one to five neurons. Furthermore, since the selection pressure coefficient of neurons is fixed between 0 and 1, choosing 0 means that it will be challenging to estimate the number of neurons, but choosing 1 will let all potential neuronal growth take place in each hidden layer. Improving the assessment indices is meant to increase the effectiveness of the GMDH algorithm. Six meta-heuristic methods with 1000 repetitions each have been iterated to select the best response. The population size, crossover rate, mutation rate, and generation size are set to 0.02, 0.7, 50, and 1000, respectively, as the input parameters for the NSGA-II algorithm. The population size, maximum number of iterations, inertia weight (w), inertia weight damping ratio (wdamp), personal learning coefficient (C1), global learning coefficient (C2), leader selection pressure (beta), and pressure removal selection (lambda) are the parameters that are set in order to process the MOPSO algorithm. These values are 50, 1000, 1, 0.95, 2, 2, 10, and 10. For the other three algorithms, the number of population and the number of generations are considered equal to 50 and 1000, respectively.

## 3 Results

In the first step, the dataset of experimental data must be known. Table 1 shows the input and output data. The input data is φ, and Temp and the output data are μ_nf_ and TC. Fig. 1 depicts the correlation value between the objective functions and the input variables. This diagram shows the effect of input variables on output. However, if this value is equal to 1, it means that the effect of that input on that output is very high. As can be seen, the effect of the first input, i.e., φ, on μ_nf_ is 0.83 and on TC is 0.92, which indicates the impact of this input on the outputs. Similarly, the second input, i.e., Temp, is −0.5 on μ_nf_ and 0.38 on TC. It can also see the changes in the input on the output with a box plot diagram. Fig. 2, Fig. 3 show changes in φ and Temp on μ_nf_ and TC of silica-alumina-MWCN/water–NF. According to Fig. 2, with the increase in φ, the value of μ_nf_ and TC of silica-alumina-MWCN/water-NFs increases, and this increase is beneficial TC, but on the other hand, it is harmful to μ_nf_. Also, in Fig. 3, with increasing Temp, the value of μ_nf_ decreases and TC increases, which is suitable for both objective functions.

**Table 1:** Data specifications.

φ (%)	Temp (°C)	μ_nf_ (cP)	TC (W/m.K)
0	20	1.307	0.586
0	30	1.23	0.603
0	40	1.163	0.618
0	50	1.103	0.631
0	60	1	0.641
0.1	20	1.98	0.641
0.1	30	1.72	0.653
0.1	40	1.55	0.668
0.1	50	1.4	0.691
0.1	60	1.24	0.703
0.2	20	2.74	0.664
0.2	30	2.11	0.681
0.2	40	1.83	0.703
0.2	50	1.54	0.729
0.2	60	1.39	0.764
0.3	20	3.3	0.701
0.3	30	2.55	0.726
0.3	40	2.12	0.739
0.3	50	1.97	0.752
0.3	60	1.73	0.775
0.4	20	3.85	0.741
0.4	30	3.26	0.765
0.4	40	2.86	0.782
0.4	50	2.29	0.798
0.4	60	2.12	0.817
0.5	20	4.76	0.765
0.5	30	3.86	0.786
0.5	40	3.26	0.799
0.5	50	2.77	0.827
0.5	60	2.4	0.856

**Fig. 2:** Correlation value between input variables and objective functions.

**Fig. 3:** Correlation value between input variables and objective functions.

**Fig. 4:** (a) Spiraling up (b) Double round and (c) Random movement.

Fig. 2 illustrates the relationship between μ_nf_ and φ and Temp deficit at various Tem. It is evident from Fig. 2 that the μ_nf_ of the fluid rises as the φ deduction increases. Conversely, Fig. 3 indicates that the μ_nf_ decreases as the Temp increases. Reasons for justifying this phenomenon are as follows.

• Brownian motion: The random motion of NPs in the base fluid is a significant factor that affects μ_nf_. This motion occurs due to continuous collisions between NPs and base fluid molecules.
• NP dispersion: When NPs are added to the base fluid, they disperse throughout the fluid and form symmetrical and larger nanoclusters. This is due to the van der Waals force between the NPs and base fluid. These nanoclusters inhibit the movement of fluid on one another, increasing μ_nf_.
• Nanostructures and their properties: Nanostructures have a super-high surface-to-volume ratio, which leads to changes in qualities such as density. Due to their ultra-small size and super-low mass, floating forces and weight lose their importance. Instead, superficial and intermolecular forces play a significant role in determining μ_nf_.
• Increased intermolecular forces: The presence of nanomaterials in the base fluid causes an increase in intermolecular forces, which in turn increases μ_nf_.

Fig. 2, Fig. 3 demonstrate a noteworthy increase in the TC of NFs as the Temp and φ increase. This trend is consistent across all Temp and φ. The rise in TC due to Temp can be attributed to Brownian motion and increased NP interaction. Conversely, an increase in φ results in a greater number of suspended NPs, leading to an increase in φ and particle collision. This, in turn, may enhance NP interaction.

Fig. 4(a–c) shows Spiraling up Double round and Random movement. After introducing evolutionary algorithms and the GMDH algorithm, it can be used now. For this purpose, experimental points must first be predicted using the GMDH algorithm. For this purpose, to increase the accuracy of the GMDH algorithm, it is combined with meta-heuristic algorithms. These algorithms were fully introduced in the previous section. Among meta-heuristic algorithms combined with the GMDH algorithm, a superior combination with higher accuracy should be selected. For this purpose, 6 evaluation criteria were selected and these combinations were reviewed and evaluated based on these criteria. The values of these criteria for 6 combinations of evolutionary algorithms with GMDH can be seen in Table 2. According to Table 2, the best performance is related to the coupling of the GMDH ANN with the NSGA II algorithm. Fig. 5 shows the calculated MOD for the μ_nf_ function. It can be found that the maximum MOD was related to GMDH + NSGA II, GMDH + MOPSO, GMDH + MOMFO, GMDH + MOWOA, GMDH + MOGOA and GMDH + MALO algorithms is equal to −0.108, −0.2186, −0.115, −0.382, −0.1724 and −0.1577, respectively. Also, Fig. 6 shows the calculated MOD for the TC function. It can be found that the maximum MOD was related to GMDH + NSGA II, GMDH + MOPSO, GMDH + MOMFO, GMDH + MOWOA, GMDH + MOGOA and GMDH + MALO algorithms is 0.0253, 0.0247, 0.02409, 0.0256, −0.0251 and 0.365, respectively.

**Table 2:** The value of evaluation criteria for the objective function (μ_nf_ of silica-alumina-MWCN/water nanofluid).

Algorithm	R	RMSE	MAE	MSE	R^2^	MAPE
GMDH + NSGA II	0.996	0.036	0.0125	0.0013	0.99996	0.659
GMDH + MOPSO	0.99506	0.0393	0.01242	0.00154	0.99995	0.6845
GMDH + MOMFO	0.99574	0.0363	0.01277	0.00132	0.98775	0.6615
GMDH + MOWOA	0.9931	0.04882	0.01451	0.00238	0.9944	0.9027
GMDH + MOGOA	0.99565	0.03613	0.01265	0.001306	0.99983	0.69248
GMDH + MALO	0.9956	0.03737	0.012574	0.001397	0.999983	0.7055

**Fig. 5:** MOD for μ_nf_ of silica-alumina-MWCN/water nanofluid.

**Fig. 6:** MOD for TC of silica-alumina-MWCN/water nanofluid.

**Fig. 7:** Schematic of ANN neurons.

According to Table 2, Table 3 and Fig. 5, Fig. 6, the GMDH ANN coupling with NSGA II has performed better than the rest of the algorithms. After choosing the best coupling of the evolutionary algorithm with the GMDH ANN, the schematic state of the combination of neurons should be determined. Fig. 7 shows the number of layers and neurons in this network. The target of using ANNs is to develop a relationship between input and output variables. These mathematical relationships are associated with combining a pair of neurons that are combined. In this way, input variables or input neurons are combined two by two to form a set of neurons. The set of neurons is positioned in one layer. This operation is repeated until it reaches the final layer, and a single neuron or objective function is achieved in this layer. According to Fig. 7, which illustrates the schematic of the neurons, it is feasible to derive the relations between the input variables and the objective functions according to Eqs. (60), (61)).

(60) $$\mu_{nf}=2.204135849688302+7.204280129127809\times \varphi -0.046934991348675\times \mathrm{Temp}+1.940639608134548\times \varphi^{2}+4.566784843459138e-04\times {\text{Temp}}^{2}-0.091242179819800\times \mathrm{Temp}\times \varphi$$

(61) $$\mathrm{TC}=0.566020879574005+0.443475896335320\times \varphi +0.001068728703283\times \mathrm{Temp}-0.236619848795991\times \varphi^{2}+5.388621949122327e-06\times {\text{Temp}}^{2}+0.001322884073301\times \mathrm{Temp}\times \varphi$$

**Table 3:** The value of evaluation criteria for the objective function (TC of silica-alumina-MWCN/water nanofluid).

Algorithm	R	RMSE	MAE	MSE	R^2^	MAPE
GMDH + NSGA II	0.9954	0.0028	0.0009	7.8e-6	1	0.125
GMDH + MOPSO	0.9952	0.00286	0.00094	8.16e-6	0.999997	0.1294
GMDH + MOMFO	0.99511	0.002864	0.00093	8.2e-6	0.999997	0.1292
GMDH + MOWOA	0.99537	0.002809	0.000915	7.89e-6	0.999998	0.1285
GMDH + MOGOA	0.99509	0.002914	0.000948	8.49e-6	0.999999	0.13217
GMDH + MALO	0.99393	0.003198	0.000972	1.02e-5	0.999997	0.134961

These equations can be used to predict the simulation data once the governing equations between the design variables and objective functions have been established. By placing the input values in the equations, output values for the μ_nf_ are obtained. The values predicted by ANN can be compared with the simulation data. Fig. 8, Fig. 9 show the difference between experiment data and predicted data by the ANN for μ_nf_ and TC. Evolutionary algorithms use ANN-generated equations as input. The objective functions, which are the μ_nf_ and TC, which μ_nf_ must be minimized, and TC must be maximized. The issue is that it is impossible to locate a point with the highest TC and lowest μ_nf_ values. As a result, optimal points known as the Pareto front are generated by meta-heuristic algorithms using input data and equations generated by GMDH-ANN.A Pareto front, which is a collection of optimal points arranged along a line, is the optimization output of meta-heuristic algorithms. The Pareto front is generated based on the results of the GMDH-ANN type. From the Pareto optimal points, the point with the best performance for the two objective functions is then chosen. To put it another way, the state that can reduce μ_nf_ and torque in a suitable proportion is thought to be the optimal point. In Fig. 10, the Pareto fronts for two objective functions are obtained by 6 evolutionary algorithms. According to Fig. 10, the GA algorithm has the best performance in the best solution. The mutation rate, crossover rate, population size, and some generations for GA algorithm processing are set to 0.02, 0.7, 100, and 1000, respectively. Eqs. (62), (63)) are used to calculate the range of design variables and objective functions.

(62) $$\mathrm{Minimize}\;\mu_{nf}=f_{1}\left(\varphi ,\mathrm{Temp}\right)$$

(63) $$\mathrm{Maximize}\;\mathrm{TC}=f_{2}\left(\varphi ,\mathrm{Temp}\right)$$

$$\mathrm{Subjected}\;\mathrm{to}:\left\{ \begin{array}{c} 0\leq \varphi \leq 0.5\\ 20\leq Temp\leq 60 \end{array}\right.$$

**Fig. 8:** Comparison of μ_nf_ predicted by ANN with experimental data.

**Fig. 9:** Comparison of predicted TC by ANN with experimental data.

**Fig. 10:** Obtained Pareto front by six evolutionary algorithms.

Fig. 11 depicts the Pareto front created by the NSGA II algorithm to provide a set of optimal points based on the experiment points' outcomes. A Pareto front, created by coupling the ANN and NSGA II Algorithm, serves as the most precise boundary for optimal points. Fig. 11 shows the simulation points, and the Pareto front, which can be seen as the Pareto front, has determined the best and most accurate boundary for optimal data with very suitable accuracy. This means that ANN equations are well-predicted, which has a decent performance. Fig. 12 and Table 4 depict four points from the Pareto front chosen by NSGA II: A, B, C, and D. Point A has the lowest μ_nf_ and TC, which, considering that the goal is to reduce μ_nf_ and increase TC, this point is appropriate for when the user has only reduced μ_nf_ as a criterion for his work. On the other hand, point D follows the opposite of this issue, and the increase in TC is useful. Among the other two points, it seems that the middle points of these two functions are the objective function, but point B can be considered the most optimal point because the values of μ_nf_ and TC are in ideal moods. The surface graphs of these two objective functions with inputs can be seen in Fig. 13, Fig. 14.

**Fig. 11:** Pareto front created by NSGA II algorithm.

**Fig. 12:** Optimal points of the Pareto front.

**Table 4:** Optimal points of the Pareto front.

Pareto	φ (%)	Temp (°C)	μ_nf_ (cP)	TC (W/m.K)
A	0.0002	50.8772	0.9988	0.6344
B	0.1916	59.532	1.4394	0.74
C	0.3057	59.616	1.75	0.7864
D	0.49986	59.9775	2.382	0.8517

**Fig. 13:** Surface plot of inputs (φ, T) and μ_nf_.

**Fig. 14:** Surface plot of inputs (φ, T) and TC.

## 4 Conclusion

This study stands out for its use of ANNs and various evolutionary algorithms to analyze and estimate μ_nf_ and TC in silica-alumina-MWCNT/water-NFs. The innovation here lies in this unique approach, employing ANN and evolutionary algorithms to explore the significant influence of φ and Temp on μ_nf_ and TC. The study emphasizes the originality of the NSGA II algorithm, when combined with ANN and GMDH, outperforming other methods with exceptional predictive accuracy. Additionally, the use of a GA to minimize μ_nf_ and TC, and the identification of optimal conditions at points A, B, C and D, introduces a novel approach for enhancing NF performance. It is worth noting that The study focuses on a specific NF composition, which may limit the generalizability of the findings to other NFs.On the other hand, this study investigates the effects of other potentially relevant parameters, such as particle size or surface treatment, which can influence the behavior of the NF. It is hoped that this study can be used to evaluate the generalizability of the modeling approach, a wider range of NF compositions and types of particles. The results of this study show that.

• Increasing the amount of φ increases the μ_nf_ and TC of silica-alumina-MWCNT/water–NF, which is beneficial for TC, but on the other hand, it is harmful to μ_nf_.
• Increasing the Temp increases the TC of silica-alumina-MWCNT/water–NF, but on the other hand, it decreases the μ_nf_.
• The best μ_nf_ estimation performance is related to ANN GMDH coupling with the NSGA II algorithm.
• The best TC estimation performance is related to ANN GMDH coupling with the NSGA II algorithm.
• The maximum MOD of the μ_nf_ function belongs to the algorithm (GMDH + NSGA II = −0.108), and the minimum MOD belongs to the algorithm (GMDH + MALO = −0.1577).
• The maximum MOD of the TC function belongs to the algorithm (GMDH + NSGA II = −0.0253), and the minimum MOD belongs to the algorithm (GMDH + MALO = 0.365).
• The maximum Pareto front belongs to group D. In this group, the input variables (φ, Temp) were evaluated as 0.49986%, 59.9775 ^°^C respectively. Also, the value of the target functions (μ_nf_ and TC) was estimated as 2.382 cP and 0.8517 W/m.K, respectively.
• Pareto minimum front belongs to group A. In this group, the input variables (φ, Temp) were evaluated as 0.0002 % and 50.8772 °C respectively. Also, the value of the target functions (μ_nf_ and TC) was estimated as 0.9988 cP and 0.6344 W/m.K, respectively.
• Pareto optimal front belongs to group B. In this group, the input variables (φ, Temp) were evaluated as 0.1916 % and 59.532 °C respectively. Moreover, the value of the objective functions (μ_nf_ and TC) was estimated as 1.4394 cP and 0.74 W/m.K, respectively.

The authors suggest that the effect of NPs on the Nusselt number, and heat flux, be examined. Also, the effect of the type and size of the NPs should be investigated in this study.

## CRediT authorship contribution statement

**Mohammadreza Baghoolizadeh:** Formal analysis, Data curation, Conceptualization. **Dheyaa J. Jasim:** Software, Resources. **S. Mohammad Sajadi:** Supervision, Software, Conceptualization. **Reza Rostamzadeh- Renani:** Writing – original draft, Project administration. **Mohammad Rostamzadeh- Renani:** Writing – review & editing, Software, Resources. **Maboud Hekmatifar:** Validation, Project administration, Data curation, Conceptualization.

## Declaration of competing interest

The authors declare that they have no known competing financial interests or personal relationships that could have appeared to influence the work reported in this paper.
